The article "Recent Updates of Natural and Synthetic URAT1 Inhibitors and Novel Screening Methods" was published in 2021. Journal: Evid Based Complement Alternat Med.

# Recent Updates of Natural and Synthetic URAT1 Inhibitors and Novel Screening Methods

**DOI:** 10.1155/2021/5738900

**Published:** 2021-10-31

**Authors:** Ying Chen, Ruya You, Ke Wang, Yousheng Wang

**Affiliations:** ^1^Beijing Advanced Innovation Centre for Food Nutrition and Human Health, Beijing Technology and Business University (BTBU), Beijing, China; ^2^Rizhao HUAWEI Institute of Comprehensive Health Industries, Rizhao, Shandong, China; ^3^Shandong KEEPFIT Biotech. Co., Ltd., Rizhao, Shandong, China

## Abstract

Human urate anion transporter 1 (hURAT1) is responsible for the reabsorption of uric acid in the proximal renal tubules and is a promising therapeutic target for treating hyperuricemia. To mitigate the side effects of URAT1-targeted clinical agents such as benzbromarone, there is significant interest in discovering new URAT1 inhibitors and developing technology that can evaluate URAT1 inhibition. This review summarizes the methods for assay of URAT1 inhibition and the progress on the discovery of natural and synthetic URAT1 inhibitors in the past five years.

## 1. Introduction

Uric acid is the final product of purine metabolism in the human body [1, 2]. In recent years, more people suffer from an unbalanced urate metabolism [3]. Hyperuricemia is characterized by insufficient excretion and the overproduction of uric acid [4] and is defined as serum uric acid concentration of >408 *μ*mol/L or 6.8 mg/dL [5]. The primary clinical characteristic of hyperuricemia is gout [6], which is a common and complex form of arthritis caused by the deposition of monosodium urate crystals in the peripheral joints and surrounding tissues. Gout prevalence ranges from 2.7% to 6.7% in Western countries and from 0.1% to 10% globally, and increases from 0.03% to 0.6% every year [3, 7]. Additionally, hyperuricemia is associated with other diseases, including chronic kidney dysfunction [8, 9], hyperlipidemia [10], hypertension [11], coronary heart disease [12], diabetes [13], and vascular disease [14, 15].

There are currently three treatments for hyperuricemia: reduction of urate production, increase in urate excretion, and decomposition of urate. Statistics indicate that 90% of hyperuricemia cases are due to impaired renal uric acid excretion and that only 10% are due to excessive production of uric acid [16]. The kidneys and intestines play a major role in uric acid excretion, with more than 70% of urate excretion taking place in the renal pathway. As such, the development of reagents for increasing uric acid excretion has significant therapeutic potential.

Human urate transporter 1 (hURAT1) is a transmembrane protein that consists of 555 amino acids and belongs to the organic anion transporters (OAT) family. URAT1 is expressed on the luminal side of the proximal renal tubule [17] and regulates the absorption of uric acid from the renal tubule to the epithelial cells [18]. As urate is eliminated from the kidneys, approximately 90% of the urate filtered by the glomeruli is reabsorbed back into the bloodstream and only 10% is excreted by the kidneys. The uric acid reabsorption process is primarily controlled by URAT1 and is particularly important to hyperuricemia. Inhibition of URAT1 is currently the main treatment for urate-lowering therapy, in addition to pills such as allopurinol and febuxostat, which block xanthine oxidase (XO) [19, 20]. Considering 90% of hyperuricemia cases are due to reduced renal uric acid excretion, the inhibition of URAT1 over XO could be a better approach to treating gout [21].

The article "Recent Updates of Natural and Synthetic URAT1 Inhibitors and Novel Screening Methods" was published in 2021. Journal: Evid Based Complement Alternat Med.

URAT1 inhibitory drugs currently approved for use in clinical settings include probenecid, benzbromarone, sulfinpyrazone, and lesinurad (Figure 1) [22–24]. However, these medicines have side effects and some degree of toxicity [25]. Probenecid can induce rash, gastrointestinal tract irritation, hypersensitivity, and hemolytic anemia [22]; benzbromarone results in serious hepatotoxicity and bone marrow suppression [26]; sulfinpyrazone can cause nausea, vomiting, abdominal pain, diarrhea, anemia, and skin rashes [27]; lesinurad has dose-dependent nephrotoxicity and can cause adverse cardiovascular events [28]. The use of URAT1 inhibitors is not recommended in patients with severe renal failure, urate kidney stones, or blood dyscrasias [25].

While xanthine oxidase inhibition is still the primary therapy for gout, it can also have serious adverse effects, such as skin rashes, hepatitis, fever, Stevens–Johnson syndrome, nephropathy, fatal liver necrosis, allergic reactions, and cardiovascular events. As such, alternative medicines with fewer side effects are needed to treat this disorder [29–31].

Considering these challenges, there is a need for alternative medicines with fewer side effects, and new therapies are needed for patients who cannot sufficiently reduce urate with current therapies. As such, there is an urgent need to discover effective and safe compounds targeting URAT1 to lower serum uric acid [32] and to develop novel techniques validating URAT1 inhibitors. This study summarizes natural and synthetic URAT1 inhibitors in the past five years. Compared with a recently published review [33], this paper outlines the chemical structures, inhibitory effects, and evaluation methods of natural inhibitors in further detail. For synthetic URAT1 inhibitors, we demonstrate different parent structures including lesinurad, verinurad, and febuxostat derivatives, displayed with both *in vitro* and *in vivo* data. We also describe classical and recent methods for evaluating URAT1 inhibitors.

The article "Recent Updates of Natural and Synthetic URAT1 Inhibitors and Novel Screening Methods" was published in 2021. Journal: Evid Based Complement Alternat Med.

## 2. Materials and Methods

This review covers the literature published in the last five years and focuses on the most relevant studies assessing cell-based *in vitro* approaches for evaluating URAT1 inhibition and novel URAT1 inhibitors. The inhibitors are organized according to the origin of the compounds (natural and synthetic) and their chemical structures. The structures of specific compounds with promising results are presented in the figures. All studies were retrieved from the following databases: Web of Science, PubMed, Scopus, and CNKI. The following keywords were used: “URAT1 inhibitors,” “hyperuricemia,” “screening methods,” “and uric acid.” The chemical structures in this article were created by ChemDraw.

## 3. Results

### 3.1. Recent Development of URAT1 Inhibitors

#### 3.1.1. Natural Compounds with URAT1 Inhibitory Activity

Natural products have received significant attention for their urate-lowering potential [34, 35], particularly phenolic compounds, terpenes, and fatty acids, all of which are reported to have antihyperuricemic activity.

*(1) Phenolic Compounds and Analogues*. Toyoda et al. [36] evaluated several flavonoids isolated from *Citrus* fruits and found that naringenin (compound 1) (IC_50_ = 16.1 *μ*M), hesperetin (compound 2) (IC_50_ = 25.7 *μ*M), and nobiletin (compound 3) (IC_50_ = 17.6 *μ*M) (Figure 2) displayed substantial URAT1 inhibitory activities with negligible cytotoxicity. The three compounds have also been studied as XO inhibitors [37] and the IC_50_ value of hesperetin is 16.5 *μ*M. However, naringenin and nobiletin have IC_50_ values exceeding 100 *μ*M, indicating that these two affect URAT1 more than XO. Some *in vivo* studies also supported their urate-lowering effects [38–40]. The oral administration of the glycon of naringenin (100 mg/kg) effectively reduced serum uric acid levels by 89% in potassium oxonate (PO-) induced hyperuricemic mice, while the positive drug allopurinol showed a 156% reduction in serum uric acid [40]. The oral administration of orange juice (5 mL/kg) and hesperetin (5 mg/kg) significantly reduced the serum uric acid in PO-induced hyperuricemia rats by 38.76% and 24.93%, respectively, while allopurinol significantly decreased by 124%. The dominant flavonoids in orange juice are hesperidin and narirutin, which are hydrolyzed to hesperetin and naringenin in the colon [38]. Citrus depressa extracts (25 mL/kg) containing nobiletin also exhibited uricosuric effects in hyperuricemia model mice, with reductions in serum uric acid levels of 22.7% compared to the PO model group [39].

The article "Recent Updates of Natural and Synthetic URAT1 Inhibitors and Novel Screening Methods" was published in 2021. Journal: Evid Based Complement Alternat Med.

Another flavonoid, baicalein (compound 4) (Figure 2), was shown by Chen et al. [41] to noncompetitively inhibit URAT1 in a dose-dependent manner with IC_50_ of 31.6 *μ*M. *In vivo* animal studies have demonstrated that 200 mg/kg baicalein can significantly lower urate levels in PO-induced hyperuricemia mice by elevating urate excretion. Docking analysis and site mutation indicate that baicalein interacts with Ser35 and Phe241 of URAT1. Baicalein was also reported to exhibit liver and kidney protection without toxicity [42, 43].

Curcumin (compound 5) (Figure 2) is a polyphenolic compound and has been reported to have uricosuric activity and URAT1 inhibition [CN101181249]. Twenty-two *α*, *β*-unsaturated cyclohexanone and cyclopentanone analogs of curcumin were later synthesized and demonstrated a remarkable antihyperuricemia effect [44]. Among them, **4d** (compound 6) (Figure 2) inhibits both URAT1 and XO. It inhibits 38.2% of URAT1 activity at 100 *μ*M, compared with 42.5% inhibition of benzbromarone at the same concentration.

To discover novel compounds for hyperuricemia, 107 crude products were screened by uric acid uptake assays on URAT1-HEK293/PDZK1 cells [45]. Of them, the MeOH extract from Cnidii Monnieris Fructus exhibited the highest inhibitory effect. Osthol (compound 7) (Figure 2) was identified as the active compound in the extract, which noncompetitively inhibits URAT1 with an IC_50_ of 78.8 *μ*M and is compatible with IC_50_ = 42 *μ*M of probenecid. *In vitro* studies demonstrated that osthol <100 *μ*M has no cytotoxicity in HEK293/PDZK1 cells. The authors also compared the URAT1 inhibition of different coumarins and found that only compounds with a prenyl group at the 8-position of osthol and osthenol (compound 8) displayed URAT1 inhibitory effects at 100 *μ*M, suggesting the important role for this substitution in URAT1 inhibition.

BDEO (compound 9) (Figure 2) is a deoxybenzoins oxime analog and has a structure similar to flavonoids. Its role as a dual inhibitor for lowering urate has been studied, and it is found that it blocked the uptake of uric acid in URAT1-293T cells (*K*_*i*_ = 0.14 *μ*M) in a noncompetitive manner and inhibited XO activity (IC_50_ = 3.3 *μ*M). *In vivo* studies demonstrated that BDEO at 5 mg/kg significantly decreased serum urate in PO-induced hyperuricemia mice and exhibited a nontoxic, dose-dependent effect. The administration of 20 mg/kg BDEO has effects comparable to allopurinol or benzbromarone at 10 mg/kg [46].

*(2) Terpenes*. Dioscin (compound 10) (Figure 3) was discovered to have weak inhibitory activity on XO in an earlier study [47] and also shows antihyperuricemic effects in animal models [48–50]. Zhang et al. explored the metabolites of dioscin and identified tigogenin (compound 11) (Figure 3) as a URAT1 inhibitor. An *in vitro* uric acid uptake assay demonstrated that only 10 *μ*M tigogenin could significantly inhibit URAT1 function and could dramatically reduce uric acid uptake by 40% at 100 *μ*M [48].

The article "Recent Updates of Natural and Synthetic URAT1 Inhibitors and Novel Screening Methods" was published in 2021. Journal: Evid Based Complement Alternat Med.

Bao et al. claimed that four quassinoids (13*β*, 18-dihydroeurycomanol (compound 12), △^4,5^,14- hydroxyglaucarubol (compound 13), 13*β*, 21-dihydroxyeurycomanol (compound 14), and eurycomanol (compound 15)) (Figure 3) from the *Eurycoma longifolia* stem 70% ethanol extract (EL) possessed URAT1 inhibitory activities at 50 *μ*M. The chemical structures of these four compounds indicate that they belong to eurycomanol type quassinoids. The EL showed the uric-lowering effect in PO-induced hyperuricemic mice and that eurycomanol significantly reduced serum uric acid levels at 20 mg/kg [51].

Additionally, alpinia oxyphylla seed ethanol extract (AE) displays strong URAT1 inhibitory activity. Its URAT1 inhibitory effect at 100 *μ*g/mL is comparable with that of benzbromarone (100 *μ*M), as shown by the uric uptake assay in hURAT1-expressing oocytes, in which only 1 *μ*g/mL AE significantly inhibit URAT1 function. UPLC analysis revealed nootkatone (compound 16) (Figure 3) as the primary bioactive compound in the extract, while *in vivo* administration of 100 mg/kg nootkatone significantly reduced serum uric acid in PO-induced hyperuricemic rats [52].

*(3) Fatty Acids*. It is well established that fatty acids (FAs) influence a range of metabolic and inflammatory diseases [53, 54] and cancer [55]. A recent study demonstrated the relationship between FAs and hyperuricemia: of 25 FAs tested *in vitro* [56], nine unsaturated FAs exhibited URAT1 inhibitory effects at 100 *μ*M, but no saturated FAs showed any effects. In particular, three long-chain unsaturated FAs exhibited strong URAT1 inhibitory effects: eicosapentaenoic acid (EPA) (compound 17) (Figure 4), *α*-linolenic acid (ALA) (compound 18) (Figure 4), and docosahexaenoic acid (DHA) (compound 19) (Figure 4), which had IC_50_ values of 6.0, 14.2, and 15.2 *μ*M, respectively. This study could lead to a new kind of URAT1 inhibitor, though the interaction between FAs and URAT1 requires additional study.

#### 3.1.2. Synthetic Compounds

*(1) Lesinurad Analogues*. Lesinurad (Figure 1) is a selective inhibitor of URAT1 and OAT4 for uric acid reabsorption, though it also displays adverse nephrotoxic effects [25]. Lesinurad is considered a scaffold compound for discovering inhibitors with reduced side effects and improved activities.

The article "Recent Updates of Natural and Synthetic URAT1 Inhibitors and Novel Screening Methods" was published in 2021. Journal: Evid Based Complement Alternat Med.

Zhao et al. [57] found that the 1-cyclopropylnaphthalene core with side chains of methyl (or dimethyl) substitution and carboxylic acid is important for lowering uric acid levels. 1H-Imidazole [4,5-b]pyridine derivative **44** (compound 20) (Figure 5) exhibited the most potent URAT1 inhibitory activity (IC_50_ = 1.6 *μ*M in comparison with 13.2 *μ*M of lesinurad). They also reported a dual inhibitor **83** (compound 21) (Figure 5) targeting both URAT1 (IC_50_ = 4.2 *μ*M) and glucose transporter 9 (GLUT9) (IC_50_ = 31.7 *μ*M), which could account for it having the best urate-lowering effect among all compounds tested.

Nineteen bioisosteres of lesinurad were designed and prepared by Wu et al. [58], and two rounds of structure-activity relationship (SAR) exploration revealed a novel, highly active URAT1 inhibitor **1g** (compound 22) (Figure 5), which contains an N-(pyridin-3-yl) sulfonamide moiety. URAT1-mediated urate transport assay demonstrated that **1g** exhibits >200-fold URAT1 inhibition (IC_50_ = 0.032 *μ*M) to lesinurad (IC_50_ = 7.2 *μ*M).

Wu et al. [59] designed and synthesized a imidazole analog of lesinurad, named LUM (2(5-bromo-1(4-cyclopylnaphthalen-1H-imidazol-2-ylthio) acetate) (compound 23) (Figure 5). The IC_50_ value of LUM for URAT1 is 3.2 *μ*M, which is significantly more potent than lesinurad (IC_50_ = 65.5 *μ*M). Oral administration of 40 mg/kg LUM produced a urate-lowering effect comparable with that observed by 80 mg/kg lesinurad in PO-induced hyperuricemic rats, suggesting that LUM is more effective than lesinurad in *in vivo* experiments. However, *in vitro* cytotoxicity experiments found cytotoxicity beginning with 50 *μ*M LUM, while 400 *μ*M lesinurad significantly affected cell viability. Therefore, although LUM has better antihyperuricemia properties, its safety and tolerability must be improved.

Another active URAT1 inhibitor **1c** (IC_50_ = 0.231 *μ*M) (compound 24) was discovered in an earlier investigation and possesses a CH_2_ group between the triazole and naphthalene rings of lesinurad (Figure 5) [60]. The authors subsequently performed four rounds of SAR exploration of this flexible naphthyltriazolylmethane skeleton and discovered two compounds of **1j** (sodium 2-((5-bromo-4-((4-n-propylnaphth-1-yl)methyl)-4H-1,2,4-triazol-3-yl)thio)acetate) (compound 25) and **1m** (sodium 2-((5-bromo-4-((4-bromonaphth-1-yl)methyl)-4H-1,2,4-triazol-3-yl)thio)acetate) (compound 26) (Figure 5) as effective URAT1 inhibitors. The IC_50_ values of **1j** and **1m** against URAT1 are 0.092 *μ*M and 0.094 *μ*M, respectively. The authors also found several key points by the SAR analysis; first, the 5-position of the 1, 2, 4-triazole ring must be a halogen atom; second, there must be no substitution on the *α*-position acetate; third, the inhibitory activity of URAT1 is enhanced increase as the space volume of (cyclic) alkyl substituents increases [61].

*(2) Other Synthetic Compounds*. CDER167 (compound 27) is an RDEA3170 (compound 28) derivative with the insertion of methylene between the naphthalene and pyridine of RDEA3170 (Figure 6). It is described as a dual inhibitor of both URAT1 and GLUT9, with IC_50_ values of 2.1 *μ*M and 91.6 *μ*M, respectively. Compared to the parent RDEA3170, CDER167 possesses similar inhibition on URAT1, though RDEA3170 shows no inhibition of GLUT9. An *in vivo* study confirmed the safety of CDER167 and that it is more bioavailable than RDEA3170 [62].

The article "Recent Updates of Natural and Synthetic URAT1 Inhibitors and Novel Screening Methods" was published in 2021. Journal: Evid Based Complement Alternat Med.

Febuxostat (Figure 6) is a nonpurine selective XO inhibitor and was approved as a first-line drug for treating hyperuricemia and gout in 2009. Zhou found that febuxostat has an inhibitory effect on URAT1 [63]. They used a fluorescence-based assay and identified the URAT1 inhibitors febuxostat and benzbromarone, which have IC_50_ values of 36.1 *μ*M and 14.3 *μ*M, respectively. As such, the authors designed and synthesized a series of “me-too” compounds using febuxostat as the lead to screen URAT1 inhibitors. They found that compound **4** (compound 29) (Figure 6) (IC_50_ value = 10.8 *μ*M) exhibits a similar URAT1 inhibitory effect as benzbromarone [64].

### 3.2. Technical Methods for Validation of Inhibitors

Various experimental methods have been used to evaluate URAT1 inhibition. Most research uses *in vitro* models for cell-based approaches (Table 1). To our knowledge, there is currently no *in vivo* model that directly evaluates URAT1 inhibition. Many studies focus on URAT1 inhibition expression in the kidneys, but there is a lack of evidence for direct interaction. Therefore, hyperuricemia animal models are used to verify the uric-lowering effect and safety of inhibitors [65]. In this review, we focus on the *in vitro* approaches to evaluating URAT1 inhibition.

#### 3.2.1. Radioisotope-Labeled Uric Acid Uptake Assays

The radioactive ^14^C-labeling method is the most popular method of quantitatively evaluating the URAT1 function (Figure 7A). This method directly reveals the uric acid transportation by URAT1 and was established when this protein was first identified [17]. In this assay, the following cell lines are typically used for URAT1-overexpression: *Xenopus laevis* Oocytes, human epithelial kidney cell, and MDCK cells. When using oocytes, hURAT1-cRNA must be synthesized, injected into the cells, and incubated for 2-3 days. The oocytes are then transferred to a Cl^−^-free solution containing [^14^C] uric acid to initiate the uptake of uric acid, while the radioactivity in the oocytes is determined by a liquid scintillation counter [71], considering that the oocyte cell model is complicated and the renal localization of URAT1, kidney cell HEK293, or MDCK cells have been used in recent years to express hURAT1 [67, 68]. In this model, the URAT1-expressing plasmid is transiently transfected into cells for 1-2 day protein expression, and the cells are then assayed for [^14^C] uric acid uptake at certain time points (20 s, 5 min, 10 min) [21, 76]. For example, for the inhibition of URAT1 by fatty acids, only 20 s of incubation is needed for uric acid uptake, which helps exclude the impact of fatty acids on the plasma membrane [56]. This method is easy, convenient, and quick. Some studies use hURAT1 stably expressed HEK293 or MDCK cells to obtain a persistent and stable model to evaluate URAT1 inhibitors [48, 68, 69].

The article "Recent Updates of Natural and Synthetic URAT1 Inhibitors and Novel Screening Methods" was published in 2021. Journal: Evid Based Complement Alternat Med.

Radioisotope-labeled uric acid uptake assays have been widely used to screen URAT1 inhibitors with high sensitivity and are capable of measuring the IC_50_ of these inhibitors (Figure 8). However, using radioisotopes could be restricted in some laboratories and it is costly to use.

#### 3.2.2. Chromatography-Based Approach

An ultra performance liquid chromatography (UPLC) method is used for nonradioactive uric acid transport assay to detect the uric acid contents of URAT1-expressing cells. UPLC requires a relatively large amount of uric acid (0.09 *μ*M) and is limited to a maximum concentration of 0.18 *μ*M [77], meaning this method depends on extracellular and intracellular concentrations of uric acid, limiting its practical use.

LC-MS/MS is an analysis used in highly selective and sensitive *in vitro* models of URAT1 inhibition [70] (Figure 7B). Similar to other cell-based methods, hURAT1-expressing cells are incubated with non-radioactive uric acid and the test compounds. The uric acid in the cell is then released and detected via LC-MS/MS. This method is unique in that it uses isotope-labeled 1,3-15N_2_ uric acid as an internal standard, which sets the limit of detection (LOD) of uric acid at 50 nM and the limit of quantitation (LOQ) at 200 nM. This approach demonstrates a highly selective and sensitive method of assessing intracellular uric acid and provides a suitable model for the *in vitro* evaluation of drug candidates targeting URAT1.

#### 3.2.3. Fluorescence Method

Fluorescent substance 6-carboxyfluorescein (not uric acid) is used as the substrate for URAT1-mediated transportation [64] (Figure 7C). In stably overexpressed hURAT1-HEK293T cells, 6-carboxyfluorescein is selectively transported by URAT1, while the transport is time-dependent and saturable (*K*_*m*_ = 239.5 *μ*M). In this method, the cells are incubated with a fluorescent substrate for one hour, after which the cells are lysed and assayed using a microplate reader. It is an economical, environmentally friendly, and convenient approach for screening URAT1 inhibitors *in vitro*. However, because of the low affinity of 6-carboxyfluorescein, the IC_50_ values of benzbromarone and lesinurad against URAT1 measured by this method could be 100 times greater than the radioactive methods, meaning that a high concentration of compounds is required to produce the fluorescence signal. The fluorescence method has the advantages of high throughput and easy quantitative analysis and is widely used to detect *in vitro* activity in recent years [78–80]. The primary disadvantage of this approach is its low sensitivity, making the identification of strong fluorescence substrates a priority.

The article "Recent Updates of Natural and Synthetic URAT1 Inhibitors and Novel Screening Methods" was published in 2021. Journal: Evid Based Complement Alternat Med.

#### 3.2.4. URAT1 Direct Binding Assay

A URAT1 binding assay was developed to identify the interactions between the proteins and inhibitors [67]. It is a similar procedure to the uric acid uptake assay, where URAT1 is first expressed in cells and URAT-enriched cell membranes are then isolated by two steps of centrifugation. The cell membranes are incubated with a radiolabeled high-affinity URAT1 inhibitor probe (e.g., ^3^H-RDEA3170) in the presence and absence of candidate compounds. If the candidate interacts with URAT1 at the same binding site of the radiolabeled probe, the intramembrane accumulated probes will be displaced or its binding to hURAT1 will be weakened [21]. This assay has identified some URAT1 inhibitors, including benzbromarone, sulfinpyrazone, probenecid, and lesinurad. Notably, this assay relies on the same binding site of inhibitors and probes and is ineffective for molecules that bind to other URAT1 sites. As such, this binding assay provides a tool for characterizing the molecular interactions of compounds with URAT1 and provides additional validation of new inhibitors.

## 4. Conclusions

URAT1 is a proven key target for promoting uric acid excretion; however, current URAT1 inhibitors have serious side effects. In recent years, many new URAT1 inhibitors have been described and this review summarizes key and novel experimental approaches that contribute to screening URAT1 inhibitors and help validate the urate-lowering effect. Radioisotope-labeled uric acid uptake assays are classical methods of validating URAT1 inhibitors. Given the disadvantages of the radioisotope method, novel identification methods have emerged in recent years. This includes nonradioactive isotope-LC-MS/MS and fluorescence detection, both of which could help explore novel URAT1 inhibitors. However, the sensitivity and efficiency of these methods must be optimized. We also summarized current progress relating to URAT1 inhibitor discovery, including natural products and synthetic compounds. Phenolic compounds are the primary category of natural URAT1 inhibitors, while synthetic inhibitors often use lesinurad as the lead scaffold. This review also demonstrates that many compounds, such as compounds 9, 21, and 27, have dual inhibitory effects on URAT1 and XO or GLUT9, which showed an excellent urate-lowering effect with more safety. Therefore, developing dual inhibitors for urate-lowering therapy is a promising area of research, though inhibition mechanisms, pharmacokinetics, and the safety of the novel URAT1 inhibitors all require further study.

The article "Recent Updates of Natural and Synthetic URAT1 Inhibitors and Novel Screening Methods" was published in 2021. Journal: Evid Based Complement Alternat Med.

## Figures and Tables

**Figure 1:** Approved URAT1 inhibitors.

**Figure 2:** Chemical structures of phenolic compounds possessed URAT1 inhibitory activities.

**Figure 3:** Chemical structures of terpenes compounds possessed URAT1 inhibitory activities.

**Figure 4:** Chemical structures of fatty acids possessed URAT1 inhibitory activities.

**Figure 5:** Structures of lesinurad synthetic derivatives with URAT1 inhibitory activity.

**Figure 6:** Structures of other synthetic derivatives with URAT1 inhibitory activity.

**Figure 7:** Schematic illustrations of cell-based methods for evaluation of URAT1 inhibitors. A: radioisotope-labeled uric acid uptake assay; B: chromatography-based approach, IS: internal standard; C: fluorescence detection method.

**Figure 8:** Structures of the URAT1 inhibitors shown in Table 1.

**Table 1:** Cell-based methods for validation of URAT1 inhibitors.

Authors	Cell model	Validation method	Compound
Toyoda et al. [36]; Saito et al. [56]	URAT1 wild type in pEGFP-C1 vector was transiently transfected into HEK293A	Radioisotope-labeled uric acid uptake assays	1; 2; 3; 17; 18; 19
Wu et al. [58]; Zhang et al. [61]	HEK293 cells stably expressing hURAT1	Radioisotope-labeled uric acid uptake assays	22; 25; 24
Zhang et al. [48]	Stably hURAT1-transfected HEK293 cells	Radioisotope-labeled uric acid uptake assays	10
Yang et al. [66]	pCMV/neo-URAT1 was stably transfected into HE-K293 cells	Radioisotope-labeled uric acid uptake assays	32; 33
Ao et al. [44]	HEK293 cells were transiently transfected with URAT1 plasmid	Radioisotope-labeled uric acid uptake assays	6
Bao et al. [51]	HEK293 T cells stably expressing hURAT1 by virus transfect	UPLC	28
Tan et al. [21]	hURAT1 was subcloned into pCMV6/neo vector and transiently transfected into HEK293T cells	Radioisotope-labeled uric acid uptake assays	28
Chen et al. [41]	hURAT1 was subcloned into pcDNA3.1(+) and transiently transfected into HEK293T cells	Radioisotope-labeled uric acid uptake assays	4
Zhao et al. [57]	hURAT1 was subcloned into pcDNA3.1(+)-EGFP-vector and transiently transfected into HEK293T	Radioisotope-labeled uric acid uptake assays	20
Zhou et al. [64]	hURAT1 was subcloned into pCMV vector and stably expressed in HEK293T	Fluorescence detection method (6-CFL as the fluorescent substrate)	29
Tan et al. [67]	pCMV6/neo-hURAT1 was transiently transfected into HEK293T	URAT1 direct binding assay	—
Tashiro et al. [45]	hURAT1 was subcloned into pCMV-SPORT6 vector and transiently transfected into HEK293/PDZK1 cells	Radioisotope-labeled uric acid uptake assays	7
Wu et al. [59]	MDCK cells stably expressing hURAT1	Radioisotope-labeled uric acid uptake assays	23
Shin et al. [68]	MDCK cells transfected with pcDNA3.1-hURAT1	Radioisotope-labeled uric acid uptake assays	Benzbromarone; 30; 31
Chen et al. [69]	Lentivirus vectors carrying hURAT1 were constructed and stably expressed in MDCK cells	Radioisotope-labeled uric acid uptake assays	Benzbromarone;
Probenecid			
Sun et al. [70]	Lentivirus vectors carrying hURAT1 were constructed and stably expressed in MDCK cells	LC-MS/MS	Benzbromarone
Lee et al. [52]	Capped URAT1 cRNA was injected into *Xenopus* oocytes	Radioisotope-labeled uric acid uptake assays	*Alpinia oxyphylla* seed extract
Wempe et al. [71]	Defolliculated *Xenopus* oocytes were injected with capped URAT1 cRNA	Radioisotope-labeled uric acid uptake assays	34
Nakamura et al. [72]	Defolliculated *Xenopus* oocytes were injected with hURAT1 cRNA	Radioisotope-labeled uric acid uptake assays	Irbesartan
Iwanaga et al. [73] Iwanaga et al. [74]	URAT1 cRNA was injected into *Xenopus* oocytes	Radioisotope-labeled uric acid uptake assays	Losartan, pratosartan, benzbromarone
Lee et al. [75]	Capped URAT1 cRNA was injected into *Xenopus laevis* oocytes	Radioisotope-labeled uric acid uptake assays	Keishibukuryogan; shakuyakukanzoto

The article "Recent Updates of Natural and Synthetic URAT1 Inhibitors and Novel Screening Methods" was published in 2021. Journal: Evid Based Complement Alternat Med.

## Data Availability

The data used in the current study are included within this article.
